The article "Comparison of spring characteristics of titanium-molybdenum alloy and stainless steel" was retracted in 2018. Reasons: no approval from an author; concerns about the authorship.

# Comparison of spring characteristics of titanium-molybdenum alloy and stainless steel

**DOI:** 10.4317/jced.53274

**Published:** 2017-01-01

**Authors:** Ahmad Sheibaninia, Anahita Salehi, Armen Asatourian

**Affiliations:** 1 DDS, MS, Associate Professor, Fellowship of Orthosurgery, Department of Orthodontic, Islamic Azad University, Dental School, Tehran Branch, Tehran, Iran; 2 DDS, MS, Private Practice, UAE; 3 DDS, Clinical instructor, Angiogenesis and Regenerative Group, Dr. H. Afsar Lajevardi Research Cluster, Shiraz, Iran

## Abstract

**Background:**

Titanium-molybdenum alloy (TMA) and stainless steel (SS) wires are commonly used in orthodontics as arch-wires for tooth movement. However, plastic deformation phenomenon in these arch-wires seems to be a major concern among orthodontists. This study aimed to compare the mechanical properties of TMA and SS wires with different dimensions.

**Material and Methods:**

Seventy-two wire samples (36 TMA and 36 SS) of three different sizes (19×25, 17×25 and 16×22) were analyzed *in vitro*, with 12 samples in each group. Various mechanical properties of the wires, including spring-back, bending moment and stiffness were determined using a universal testing machine. Student’s t-test showed statistically significant differences in the mean values of all the groups. In addition, metallographic comparison of SS and TMA wires was conducted under an optical microscope.

**Results:**

The degree of stiffness of 16×22-sized SS and TMA springs was found to be 12±2 and 5±0.4, respectively, while the bending moment was estimated to be 1927±352 (gm-mm) and 932±16 (gm-mm), respectively; the spring-back index was determined to be 0.61±0.2 and 0.4±.09, respectively (*p*<0.001). There were no statistically significant differences in spring-back index in larger dimensions of the wires.

**Conclusions:**

Systematic analysis indicated that springs made of TMA were superior compared to those made of SS. Although both from economic and functionality viewpoints the use of TMA is suggested, further clinical investigations are recommended.

** Key words:**Bending moment, optical microscope, spring-back, stainless steel, stiffness, titanium‒molybdenum alloy.

## Introduction

In orthodontics, tooth movements are achieved by the forces developed in the deformed wire, which are transmitted to the teeth through fixed or removable appliances. The appliance is continuously subjected to masticatory forces, and hence the wire must be sufficiently resilient to resist permanent deformation and thermocycling and maintain its activation (1,2). One of the challenges of fixed orthodontic appliances is uneven arch-wire surfaces that cause friction between the wire and bracket in sliding mechanisms (3). An uneven arch-wire surface, following corrosion, becomes a site for plaque accumulation and a source for bacterial growth (4). Stainless steel (SS) wires are one solution because they have a smoother surface compared to titanium‒molybdenum alloy (TMA) and nickel‒titanium alloy (NiTi) (5,6) and may different biological characteristics (7-10); however, if they are deformed, their steel wires will also have uneven outer surfaces.

Although the properties required in an orthodontic wire vary depending on its application, generally the desirable mechanical characteristics are high spring-back, low stiffness, good formability and low friction (11,12). Stainless steel arch-wire is one of the most widely used materials in orthodontics due to its good formability, greater ease of welding and good corrosion resistance (13,14). SS wires are smooth wires with low friction and spring-back values, which are considered a reference material for comparing the characteristics of other types of orthodontic wire alloys (6). This drawback of SS led to the popularization of TMA with superelasticity, making it highly resistant to plastic deformation (15). It has been reported that TMA wires also exhibit exceptional advantages similar to SS wires, in addition to being more resistant to deformation than SS (11).

It is known that the biocompatibility of TMA materials is mainly due to surface-passive film (16,17). The TiO2-based passive film on the surface of wires provides a good measure of biocompatibility (18); furthermore, TMA is described as having an excellent balance of properties, including high spring-back, low stiffness, high formability and the ability of direct welding (11,12,19,20). Also they are considered superior to SS wires due to their favorable functional and aesthetic effects (21). However, a major drawback of TMA is its high coefficient of friction (6,22). The limitation of these types of studies was the difficulty associated with the experimental research on the smooth wires (23,24). Overall, the development of titanium-based arch-wires made it possible to use larger wires since they offer similar ranges of forces but better bracket engagement.

Meanwhile, in most cases, it is necessary to re-form wires into springs in order to apply force on the tooth (25). Therefore, it is necessary to analyze whether the metal used is capable of performing the desired functionality better than SS. To the best of our knowledge, such an analysis has not yet been reported in the literature. Therefore, this study was conducted to compare the stiffness, bending moment and spring-back properties of TMA and SS wires deformed to finger springs. In addition, this study aimed to conduct a metallographic comparison of SS and TMA wires following deformation into finger springs, using optical microscopy.

## Material and Methods

Stainless steel and TMA wires were purchased from Dentaurum GmbH & Co. (Ispringen, Deutschland). A total of 72 wires (36 SS wires and 36 TMA wires) of 3 different sizes (16×22, 17×25, 19×25) were used for the study, with 12 wires in each group. The wires were made into springs by using a special plier, as shown in figure 1A,B.

**Figure 1:** A) Springs. B) Special plier. C) Samples of mounted wires, studied in different positions. D, E) Graphs of load/deflection and bending moment in degree and spring-back at yield point.

The wires were randomly selected and mechanical properties, including stiffness, bending moment and spring-back, were determined using a soft tensile and compression testing machine (DY-34 Adamel Lhomargy, France) (23). The output of the tensile machine provides the load/deflection curve, from which the stiffness, bending moment and spring-back of the springs could be extracted and compared.

The wires were made into springs of desired diameters by wrapping around the plier #139 (KNIPEX-Werk, Wuppertal, Germani), as presented in figure 1B. The length of the wire from the top of the wire to the circular center, required for providing 5-cm spring figures, was 14.625 cm for 16×22 mil wires, 14.75 cm for 17×25 mil wires, and 14.875 cm for 19×25 mil wires. Similarly, the length of the wire from the top of the wire to the spot of the wire inside the jaw was approximately 3.15 mil. The interior diameter of loop was considered to be 6 times of the round wire diameter. The equivalent round loop diameter was calculated using the following formula after the units were changed to millimeter (Fig. 2), where D (mm) was the equivalent round wire diameter and, a (mm) and b (mm) were the lengths of rectangular sides. For instance, the loop diameter for the 16×22 mil wire was calculated as follows: (Fig. 3).

**Figure 2:** Formula.

**Figure 3:** Formula.

Similarly, the loop diameter was calculated to be 3.49 mm and 3.75 mm for 17×25 mil and 19×25 mil, respectively. The internal diameter of the springs were measured with caliper.

Before examining all the wires, a pilot study was performed to acquire the best results in the current test equipment, in addition to getting familiar with the functioning of the machine. During the analysis, the loops with diameters slightly higher or lesser than the desired value, and also the loops that were under pressure during bending were omitted, as they could probably result in inappropriate bending consequences. More importantly, the wires with wider length were kept wrapped around the bar in order to maintain the bar form unchanged and safe against the wrapped wires. This could be realized by using cryotool metals that are called SPK and /or VCN 100-150, 200 and /or CK. We used the tool CK 45.

Based on the movement degree, which was obtained from the force-movement values, two graphs were drawn for each sample using Microsoft Office Excel (2010) software (Microsoft Corporation, USA), one graph for load/deflection and another for bending moment as schematically presented in figure 1D, E.

First, the vertical force of compiler and then the length added by skidding were estimated since the design is such that the force direction does not change. This increment occurred at a ratio of 1/cos θ. Bending moment was calculated through force*span length. Following that, the bending moment graph was also drawn based on the estimated degree and the values. This graph was used for estimating the spring-back at the yield point, which, according to Burstone *et al*. (26), is the most clinically used method in practice. The yield definition was used for acquiring the yield point since all the graphs had rejected the yield point and reached the ultimate. After determining the yield point, it was controlled with supervisor and the tangent of the graphs was derived. Typically, a tangent line parallel to the yield point was drawn. The point that disconnects the x-axis was estimated to be the permanent bending angle.

-Metallographic visualization

This part of study was similar to that carried out by Zorko & Rudolf (27). The springs were randomly selected. For metallographic assessment of wires, samples were selected from loop-shaped wires. Then, the samples were cold-embedded in methylmethacrylate polymer, which has no effect on physicochemical properties of the wire. Without mounting the specimens it would be difficult since wire specimens are very thin and would not remain in the required position. Samples were prepared in both cross-sectional and longitudinal sections (Fig 1C). To be examined under a microscope, the mounted samples required surface polishing and etching. Polishing was performed by rough to smooth sand papers, respectively (with moisture), followed by etching. Different etching solutions were used for TMA and SS samples. Etching material for TMA and SS are known as Kroll’s Reagent and Glycergia, respectively.

After etching, the samples were rinsed in ethanol to remove any contamination. This is particularly essential in the case of etched SS since etching material for these wires contains glycerol, which produces a greasy surface covered by corrosion products from the etching procedure. Next, the samples were rinsed in water and dried under a dryer, and then examined under an optical microscope at ×100 magnification. With sufficient etching, the samples were examined at magnifications ×50-100, ×200-500 and ×1000 (Figs. 4,5).

**Figure 4:** Stainless steel can be seen in these figures. In A and B, it was mechanically processed and then underwent annealing. In this state, elasticity of the material decreased. Yet, in samples in this study, despite mechanical processing, this structural state was not observed in orthodontic wires (magnification ×100 was used). In C, stainless steel sample at magnification ×100 is observed, and the same sample is shown at magnification ×500 in D. It should be noted that images in figures C and D were prepared from longitudinal sections of the wire. In C, austenite grains and some impure particles are seen. In D, austenite grains contain slip lines (slip bands), which are created by mechanical processing (mechanical work is imposed on the wire during production process), and there is also distribution of carbide particles. (With severe mechanical deformation, austenite state of steel wire is transformed into martensitic phase that has magnetic properties). In E, severely elongated austenite texture is seen in stainless steel, as well as mechanical processing imposed on the wire during looping (bending) (magnification ×100). In F and G, the loop is seen with magnification ×500, and also slip lines and distribution of carbide particles in elongated austenite background, which are indistinguishable. It can be seen that this state may have been caused by cold-working during production process or by mechanical work in looping wires. In H, bent stainless steel is seen at magnification ×1000. Distribution of carbide particles in austenite background, with signs of mechanical deformation are also seen (mechanical work makes wires more elastic). In I, longitudinal view of elongated stainless steel wire is seen at magnification ×100. Elongated austenite texture, carbide particles and impurities are seen in this section.

**Figure 5:** A. Straight titanium alloy wire is seen at magnification ×100, and beta-titanium grains and impurity particles are also seen. In B, again straight titanium wire is observed at magnification ×100, with solid solution of beta-titanium and α needle phase at grain boundaries. In C, the same wire is observed at magnification ×100, with coaxial β grains and α needle phase. In D, loop-shaped beta-titanium wire is seen at magnification ×100, together with elongated beta-titanium texture, distribution of α solid solution, and some signs of mechanical processing. In E, bent beta-titanium wire is observed at magnification ×1000, with coaxial β grains, but signs of mechanical processing are unclear. In F, elongated beta-titanium is seen at magnification ×50. Residual effects of mechanical deformation due to tension and full thickness of wire, as well as signs of etching are evident. In G, coaxial beta-titanium grains containing α particle are observed at magnification ×100. Despite observable effects of mechanical deformation due to tension, particles are seen in the same form as before. In H, the same wire is seen at magnification ×500, with boundaries of beta-titanium grains and α phase. Photograph shows that beta-titanium has been used in coaxial state, together with mechanically worked stainless steel samples. Mechanical processing has been carried out on beta-titanium, followed by heat treatment to remove signs of mechanical processing. However, in stainless steel, signs of mechanical processing performed were not removed, suggesting beta-titanium does not require mechanical work for elasticity (springiness). In I, beta-titanium grains and distribution of α phase are seen at magnification ×1000.

All the three indices (stiffness, bending moment, and spring-back) need to be compared two-by-two (material type). Therefore, they were statistically evaluated with t-test. Then, the differences were recorded in percentages as well.

## Results

The spring properties of different wires with different dimensions are summarized in  Table 1. The wire 16×22 SS stiffness was found to be 12±2 grf/mm, which was nearly 2.4 times that of TMA wire at the same size. Mean stiffness of 17×25 SS wire was 19±2 grf/mm, which was 2.7 times greater than that of TMA wire. Also, mean stiffness of 19×25 SS wire was 22±3 grf/mm, which was twice the stiffness of the same size of TMA wire.

**Table 1:** Spring characteristics exhibited by springs of dimension 16 x22, 17 x25 and 19 x25.

Statistical analysis showed that the stiffness, bending moment and spring-back of TMA springs were significantly lower than those of SS wires (*P*<0.001), except for spring-back of 17×25 and 19×25 (*P*>0.05).

## Discussion

During the preparation of springs from wires, the interior diameter of the loop should be made at least 6 times of the wire diameter in order to obtain the best mechanical results (28). Since the segments were rectangular in shape, the areas of the wires were calculated, and considered to be equal to the circular area with diameter D. The value, almost 6 times of the calculated wire diameter was considered as the interior diameter the of loop. In the pilot study, it was observed that when the wires were wrapped around this medium the internal diameter was approximately 0.25 mm more than the desired value. For instance, when the 16×22 mil wire was wrapped around the partial bar of diameter 3.25 mm, the inside diameter of the obtained loop was 3.5 mm, as assessed by Caliper with ±0.1-mm accuracy. In order to overcome this issue each wire was wrapped around the bar of diameter one size less than the originally used bar. For instance a bar with a 3-mm diameter was used for wrapping 16×22 mil wire.

Among experimental groups, the least stiffness was observed in 16×22 and 19×25 sizes in TMA and SS wires, respectively. TMA size 16×22 had the lowest bending moment and elasticity, while SS size 19×25 had the highest. In fact, elasticity of beta-titanium wires 16×22, 17×25, and 19×25 was 2, 2.6 and 2.16 times lower, compared to the same size SS wires, respectively.

The stiffness value calculated in the present study was somewhat different from the results of another study carried out by Kusy *et al.* (19) due to different formulae used for calculations. In another study the appliance stiffness was calculated as follows: Appliance Stiffness=Wire Stiffness × Design Stiffness Coefficient

As the appliance has been tested, the design stiffness coefficient should also be incorporated, while for the straight wire, there is no need for such a coefficient. The differences between the results of Kusy *et al.* (19) and those of the present study are expected because straight wire was used in that study, while finger springs were used in the present study. Furthermore, the processing during the production of orthodontic wires (cold work and annealing) has an important influence on their mechanical properties (29-31). The differences in stiffness values between the two studies could also be attributed to the slight differences in alloys and percentages of constituent elements, all of which can affect stiffness. Overall, the results of the current study confirmed that the stiffness of TMA alloy is lower that the SS alloy as many other researchers have reported (6,22,32,33).

According to Burstone’s study (26), the degree of maximum bending moment in all the tested wires of the same size was 2-3 times larger than that of the current study for both SS and TMA. 19×25 mil SS was reported to be 8125±50 (gmf/mm), while that of the present study was found to be 4412±514 (gmf/mm). The difference between the degree of maximum bending moment reported in Burstone’s study with that of the current study could probably be attributed to differences between the force pressure and fixture with wire in it. In addition, the wires considered in the present study were in the form of a spring with a diameter of approximately 3 mm with helix (11). On the contrary, the wires analyzed in Burstone’s study were smooth and without helix. Therefore, it is reasonable to believe that the differences between the forms and manufacturers also affects the bending moment (18). In general, it could be mentioned that the values observed in this study were comparatively similar to those reported in the literature.

In order to ensure a uniform etching and to obtain realistic and representative microstructure, the ultrasonic cleaning was performed before etching. Otherwise, samples were etched using HF-HNO3-CH3COOH, at a ratio of 2:5:5, as an etchant for better visualization of grain boundaries (27).

In most samples grain boundaries were intact and inconsistent with previous studies; also TMA samples had bright and uniform structures in term of porosity over the surface than SS samples.

The results derived from this study indicated that TMA metal is better than SS in terms of stiffness and bending moment indexes in all the dimensions. This is also true in case of spring-back index in 16×22 mil wires. However, there were no statistically significant differences in 17×25 and 19×25 wires. Literature review indicates that there are no studies available on the spring properties of TMA and SS wires in the form of finger springs. Even in studies that compared TMA and SS wires, the spring characteristics specified for the straight forms were used (19). Various studies have shown that TMA is better in all the dimensions (11), consistent with the results of the current study.

As mentioned earlier in the introduction section, smooth surface wires are used in clinical trials. However, useful changes in form should be (1-35) made to provide tooth movement (28). This is the limitation the present study did not attempt to evaluate clinically. But it is well documented that TMA has a rough surface and SS wire has a smooth surface (3,35).

In conclusion, it seems that generally the use of smaller dimensions, 16×22, is recommended. On the other hand, among all the three indices, stiffness is the most important index in which TMA performs better than SS (11). Despite the high price of TMA and welding aspects (34) compared to that of SS, the functionality of TMA is much superior than that of SS.
